# Identification of Five Immune-Related lncRNAs Predicting Survival and Tumor Microenvironment Characteristics in Breast Cancer

**DOI:** 10.1155/2021/6676692

**Published:** 2021-02-27

**Authors:** Ran Xiao, Meng Yang, Yuanyuan Tan, Rumeng Ding, Duolu Li

**Affiliations:** ^1^Department of Pharmacy, The First Affiliated Hospital of Zhengzhou University, Zhengzhou 450052, China; ^2^Department of Cardiology, The 7th People's Hospital of Zhengzhou, Zhengzhou 450006, China

## Abstract

A common cancer in females, breast cancer (BRCA) mortality has been recently reduced; however, the prognosis of BRCA patients remains poor. This study attempted to develop prognostic immune-related long noncoding RNAs (lncRNAs) for BRCA and identify the effects of these lncRNAs on the tumor microenvironment (TME). Gene expression data from The Cancer Genome Atlas (TCGA) database were collected in order to select differentially expressed lncRNAs. Immune-related lncRNAs were downloaded from the ImmLnc database, where 316 immune-related lncRNAs were identified, 12 of which were found to be significantly related to the prognosis of BRCA patients. Multivariate cox regression analysis was then applied to construct prognostic immune-related lncRNAs as the risk model, including C6orf99, LINC00987, SIAH2-AS1, LINC01010, and ELOVL2-AS1. High-risk and low-risk groups were distinguished according to the median of immune-related risk scores. Accordingly, the overall survival (OS) in the high-risk group was observed to be shorter than that in the low-risk group. qRT-PCR analysis demonstrated that lncRNA expression levels in BRCA cell lines were in basic agreement with predictions except for LINC00987. By validating numerous clinical samples, lncRNA C6orf99 was shown to be highly expressed in the advanced stage, while LINC01010 and SIAH2-AS1 decreased in the advanced T-stage and M-stage. Moreover, the expression of LINC0098 was found to be significantly decreased among the groups (>50 years old). Gene set enrichment analysis (GSEA) was applied to analyze the cancer hallmarks and immunological characteristics of the high-risk and low-risk groups. Importantly, the TIMER database demonstrated that this immune-related lncRNA risk model for breast cancer is related to the infiltration of immune cells. In conclusion, the results indicated that five immune-related lncRNAs could be used as a prognostic model and may even accelerate immunotherapy for BRCA patients.

## 1. Introduction

Breast cancer (BRCA), one of the most common cancers among women in the world, is the main cause of death in females whose incidence increases every year [1, 2]. Although advanced diagnosis and treatment protocols have greatly reduced the mortality of BRCA, pathological results and prognosis still vary among individuals due to the high heterogeneity present in BRCA patients [3]. Certain studies have recently reported that the prognosis of BRCA patients is related to immunity [4, 5]. Hence, it is necessary to ascertain novel immune predictors in order to improve the diagnosis and treatment of BRCA.

The tumor microenvironment (TME), which is composed of immune cells, mesenchymal cells, cytokines, and other molecules, is involved in the occurrence, development, and prognosis of tumors [6, 7]. Various key genetic markers can change the prognosis of BRCA patients in TME [8, 9]. Meanwhile, tumor-infiltrating lymphocytes (TILs) of TME are also key in tumor immunotherapy [10]. Recent studies have demonstrated that TILs can act as a clinicopathologic prognostic model for BRCA patients [11, 12], and increasing TIL concentration could predict the response to neoadjuvant chemotherapy in all molecular subtypes of BRCA [13].

Long noncoding RNA (lncRNA), a major type of noncoding RNA with transcripts longer than 200 nt [14], has exhibited various roles in tumor occurrence, development, and tumor immune response [15, 16]. In particular, abnormally expressed lncRNAs may act in the process of cell proliferation, apoptosis, invasion, metastasis, and epithelial-mesenchymal transition, leading to a poor prognosis [17]. For example, lncRNA HOTTIP regulates CSC-like properties by increasing the miR-148a-3p/WNT1 expression in BCSCs [18]. Additionally, lncRNA TCL6 influences immune cell infiltration and indicates worse survival in BRCA [19]. Interfered expression of lncRNA SNHG1 could inhibit the differentiation of Treg cells by regulating miR-448/IDO and affect the immune escape of BRCA [20]. Recently, studies suggest that some lncRNAs could serve as potential prognostic model in breast cancer [21, 22], but expression and clinical value of lncRNAs in breast cancer are not validated. In addition, tumor microenvironment characteristics of immune-related lncRNAs associated with BRCA prognosis remain poorly understood.

In the present study, an immune-related lncRNA (C6orf99, LINC00987, SIAH2-AS1, LINC01010, and ELOVL2-AS1) prognostic model was established through Cox regression analysis in BRCA patients. In addition, the model was found to perform well for overall survival (OS). In addition, the proposed model considered cancer hallmarks and the immune processes, which play a vital role in BRCA tumorigenesis. Subsequently, based on the Tumor IMmune Estimation Resource (TIMER) database, the proposed model was shown to be highly correlated with immune cell infiltration. In summary, an immune-related lncRNA model was successfully constructed, which has the potential to predict the prognosis of BRCA patients (Figure 1) and provide a guide for clinical diagnosis and treatment.

## 2. Materials and Methods

### 2.1. Download and Pretreatment of Data

The transcriptome RNA-sequencing data of BRCA was acquired from The Cancer Genome Atlas (TCGA) data portal (https://portal.gdc.cancer.gov/), which contains 113 nontumor tissues and 1039 BRCA tissues. We collected and extracted clinical data of patients, excluding the ones with survival data ≤ 30 days that might die of other serious diseases, such as cerebral hemorrhage, asthma, and myocardial infarction. The data was updated on July 11, 2020. Perl language (http://www.perl.org/) was used to merge RNA-seq results into matrix files. Referring to the Ensemble database (http://asia.ensembl.org/index.html), the Ensemble ID of the gene was converted into a gene symbol matrix. Differentially expressed lncRNAs were then selected based on ∣log2FC | >2, and false discovery rate (FDR) < 0.05 by R 3.5.1 software. Immune-related lncRNAs of BRCA were downloaded from the ImmLnc database [23] (http://bio-bigdata.hrbmu.edu.cn/ImmLnc). The ImmLnc dataset in this database was lncRNAs with immune pathway-related activities obtained from TCGA. However, whether the expression of these lncRNAs is different in breast cancer and normal tissues is yet to be known. By performing the above two approaches, differentially expressed immune-related lncRNAs were detected by Venn analysis.

### 2.2. Identification of Prognostic Immune-Related lncRNAs

According to the survival time and survival status of breast cancer patients in TCGA, univariate Cox regression analysis was used to screen survival-related lncRNAs with *p* < 0.001 as the criteria. 12 immune-related lncRNAs were obtained. Hazard ratio (HR) was used to specify immune-related lncRNAs into protective (HR > 1) and deleterious portions (HR < 1).

Multivariate Cox regression analysis was then used to screen out five lncRNAs from the above 12 lncRNAs in order to establish immune-related lncRNA risk models as an independent prognostic indicator (*p* < 0.05), after which the risk score for each patient was calculated based on the expression levels of lncRNAs. According to the median risk score, BRCA patients were divided into a high-risk group and a low-risk group with the following formula: risk score = Exp1 × lncRNA1 + Exp2 × lncRNA2 + ⋯+Expi × lncRNAi, where Expi was the expression value of each immune-related lncRNA in the sample and lncRNAi was the regression coefficient of the multivariate analysis model. The overall survival (OS) of patients between the high-risk and low-risk groups was compared by Kaplan-Meier survival analysis. Additionally, the relationship between immune-related lncRNAs and clinicopathologic characteristics of BRCA patients was analyzed, including stage, T-stage, N-stage, M-stage, and age, so as to investigate their relevance.

### 2.3. Role of the Five Immune-Related lncRNAs in Immunologic Features

Gene set enrichment analysis (GSEA) was performed to verify the functional phenotypic differences between the low-risk group and the high-risk group. Afterward, the gene sets of “h.all.v7.1.symbols.gmt [hallmarks] and c7.all.v7.1.symbols.gmt [Immunologic signatures]” were analyzed from the Molecular Signatures Database (MSigDB) (https://www.gsea-msigdb.org/gsea/msigdb/). Gene sets performed permutations 1000 times, and a nominal *p* < 0.05 as well as a false discovery rate < 0.05 was considered to be significant.

### 2.4. Correlation Analysis of Immune Cell Infiltration

Tumor-infiltrating immune cell data, including B cells, CD4+ T cells, CD8+ T cells, dendritic cells, macrophages, and neutrophils, were downloaded from the TIMER database (https://cistrome.shinyapps.io/timer/). Pearson correlation was designed to calculate the association of immune-related lncRNA risk scores and infiltration of 6 immune cells.

### 2.5. Statistical Analysis

Cox regression analysis and Pearson correlation analysis were applied to identify the immune-related lncRNAs. All statistical analyses were conducted using the R statistical environment with different packages (R version 3.5.1; Institute for Statistics and Mathematics, Vienna, Austria). *p* < 0.05 was considered to be significant.

### 2.6. Cell Lines and Culture Conditions

BRCA cell lines HBL-100, HTB-20, MCF-7, MDA-MB-231, and MDA-MB-468 were purchased from the cell bank of the Chinese Academy of Sciences. Cells were cultured in RPMI-1640 medium (HyClone) and supplemented with 10% fetal bovine serum (BI) at 37°C and 5% CO_2_.

### 2.7. Quantitative Real-Time Polymerase Chain Reaction (qRT-PCR)

TRIzol reagent (Invitrogen, Carlsbad, CA, USA) was used to extract the total RNA from cultured cells in order to determine the concentration and purity of RNA, which were reversely transcribed into complementary deoxyribose nucleic acids (cDNAs; PrimeScript RT Reagent; TaKaRa, Dalian, China). Using the SYBR® Premix Ex Taq™ kit (TaKaRa, Dalian, China) and StepOnePlus Real-Time PCR system (Applied Biosystems, Foster City, CA, USA), qRT-PCR was carried out. Here, the C6orf99 primers (Sangon Biotech, China) were 5′-GATGTTCCTTGGGCTGGTTGGTC-3′ (sense) and 5′-ACCTCTCCACCTGTTCTTCACTCC-3′ (antisense); LINC00987 primers (Sangon Biotech, China) were 5′-CCGCCTCTTCCACAACTTCCTTC-3′ (sense) and 5′-CAGAGTCCCTGAACTGTCGCTTTC-3′ (antisense); SIAH2-AS1 primers (Sangon Biotech, China) were 5′-GACTCCATCTCCAACCAACCAACC-3′ (sense) and 5′-CACTAGAAAGCCTTGCCCTCCATC-3′ (antisense); LINC01010 primers (Sangon Biotech, China) were 5′-GCCCAGAAGTCAAAGTCCAGCAG-3′ (sense) and 5′-AGCACCTCCTCTTCCACATCCC-3′ (antisense); ELOVL2-AS1 primers (Sangon Biotech, China) were 5′-AGAGAGCTGCCTTGCCCTTCC-3′ (sense) and 5′-AGAGTGGGTGTCTGGTGGTAAGC-3′ (antisense); and GAPDH primers (Sangon Biotech, China) were 5′-GCATCCTGGGCTACACTG-3′ (sense) and 5′-TGGTCGTTGAGGGCAAT-3′ (antisense). The 2^-*ΔΔ*Ct^ method was used to calculate the relative gene expression levels of these lncRNAs, which were normalized to the corresponding GAPDH mRNA levels.

## 3. Results

### 3.1. Acquisition of Immune-Related lncRNAs

The RNA-seq of 1039 BRCA patients and 113 normal samples was collected from TCGA. Then, the RNA-seq data of lncRNA and mRNA were separated, and the gene read counts were normalized to the trimmed mean of M values (TMM) by EdgeR. Accordingly, 1505 differentially expressed lncRNAs are shown in Figure 2(a).

According to the ImmLnc database, 3791 immune-related lncRNAs in BRCA were obtained. Next, 316 immune-related lncRNAs were selected by matching ImmLnc gene sets with differentially expressed lncRNAs in TCGA, which were named immune-related lncRNA sets (Figure 2(b)).

### 3.2. The Five Immune-Related lncRNAs Were an Independent Prognostic Factor

By conducting a univariate Cox regression analysis, 12 lncRNAs were found to be associated with prognosis, including C6orf99, MIR4435-2HG, LINC00536, AP001412.1, CBR3-AS1, SPACA6P-AS, LINC00987, SIAH2-AS1, STK4-AS1, LINC01010, LINC01235, and ELOVL2-AS1. The corresponding forest map clearly illustrated the relationships between these 12 lncRNAs as well as their prognosis (Figure 3). Through a multivariate Cox regression analysis, 5 more meaningful lncRNAs (C6orf99, LINC00987, SIAH2-AS1, LINC01010, and ELOVL2-AS1) were further screened out from the above 12 lncRNAs (Table 1), after which a prognostic immune-related lncRNA model was established, in which the BRCA samples were divided into a high-risk group and a low-risk group based on the intermediate risk score (Figure 4(a)). It was observed that the mortality rate continued to increase with the improvement of risk score (Figure 4(b)). In addition, with a rise in risk score, the expression level of C6orf99 increased, while that of LINC00987, SIAH2-AS1, LINC01010, and ELOVL2-AS1 decreased, as shown in Figure 4(c). Furthermore, Figure 5 revealed that the survival time of the high-risk group was significantly shorter than that of the low-risk group. C6orf99 demonstrated significance in luminal A and basal-like cell subtypes (MCF-7 and MDA-MB-231), while SIAH1-AS1 and ELOVL1-AS1 had a lower expression in all cell subtypes compared to the normal cell. More notably, LINC01010 had a meaningful lower expression in the luminal A cell but was overexpressed in basal-like cell subtypes (MDA-MB-231 and MDA-MB-468) (Figure 6).

In order to further investigate the relevance of immune-related lncRNAs as well as the clinicopathologic features of BRCA, the correlation of immune-related lncRNAs and clinical characteristics, such as age and various stages, was analyzed. Here, the expression of C6orf99 was observed to be enhanced, while LINC01010 and SIAH2-AS1 were opposite in the more advanced stage. However, the expression of ELOVL2-AS1 was found to be decreased in the more advanced M-stage and N-stage, while that of LINC0098 was decreased significantly when the age was more than 50 (Figure 7). In the independent risk analysis, age, stage, T-stage, N-stage, M-stage, and immune-related risk score were noted to be significantly correlated with OS in the univariate analysis (*p* < 0.05); however, only age and immune-related risk score were remarkably correlated with OS in the multivariate analysis (Table 2). The ROC curves demonstrated the accuracy of the model. Meanwhile, the AUC values of immune-related risk score, age, stage, T-stage, N-stage, and M-stage were 0.733, 0.775, 0.719, 0.709, 0.591, and 0.641, respectively (Figure 8). In brief, the obtained results demonstrated that the proposed immune-related lncRNA model served as an independent prognostic factor.

### 3.3. The Five Immune-Related lncRNAs Mediated Glycolysis, Oxidative Phosphorylation, MYC Targets, and Immunologic Characteristics

To explore the potential molecular mechanisms of the five immune-related lncRNAs in BRCA progression, GSEA was carried out between the high-risk and low-risk groups. The corresponding results of cancer hallmarks showed that glycolysis, oxidative phosphorylation, and MYC targets were activated by the five immune-related lncRNAs in the high-risk group (Figures 9(a)–9(c)). In addition, the five immune-related lncRNAs also modulated immunologic signatures, such as naive CD4 T cells, and stimulated CD4 Th1 cells, downregulated CD8 T cells, and upregulated Treg cells. (Figures 9(d)–9(f)). Hence, the five immune-related lncRNAs may be involved in immune regulation.

### 3.4. The Five Immune-Related lncRNAs Were Negatively Correlated with the Infiltration of Six Immune Cells

In regard to the five lncRNAs that were sorted out, the correlation between their risk score and the infiltration of immune cells was analyzed using the TIMER database. As shown in Figures 10(a)–10(f), the correlation values of CD4+ T cells, CD8+ T cells, B cells, dendritic cells, neutrophils, and macrophages were -0.181, -0.22, -0.061, -0.223, -0.171, and -0.220, respectively, suggesting that the infiltration of these immune cell subtypes was significantly negatively correlated with the prognosis of BRCA. Taken together, these results indicated that the five immune-related lncRNAs were associated with the infiltration of these immune cell subtypes in BRCA.

## 4. Discussion

BRCA is a highly heterogeneous malignant tumor due to its genomic and genetic diversity [24]. In recent decades, several molecular markers focusing on mRNAs or miRNAs proved helpful in optimizing therapy decision-making among BRCA patients [25]. More recently, the perturbation of the lncRNA expression was widely recognized in multiple cancer types, altering tumors [26]. lncRNAs are involved in the regulation of diversified biological functions, such as autophagy, metabolism, inflammation, and the immune response [27, 28]. In the present study, in conjunction with the considerable amount of clinical data on BRCA, five lncRNAs, including C6orf99, LINC00987, SIAH2-AS1, LINC01010, and ELOVL2-AS1, were confirmed as a prognostic model for breast cancer. Various studies have posited that LINC00987 is reduced in patients with ankylosing spondylitis [29]. LINC01010 has a significant prognostic value that suppresses cancer cell migration and invasion of lung cancer [30]. ELOVL2-AS1 was also shown to be positively correlated with the survival rate of BRCA patients and may serve as a potential diagnostic or prognostic marker [31]. Similarly, these five lncRNAs were quantitatively analyzed via conventional qRT-PCR. Accordingly, SIAH1-AS1 and ELOVL1-AS1 were found to have a lower expression in all BRCA cell lines; hence, they were featured in the proposed model. Furthermore, LINC01010 and C6orf99 exhibited meaningful properties in basal-like cell subtypes, and their high expressions better predicted the more aggressive form of breast cancer, such as basal-like BRCA.

Contrary to luminal A BRCA subtype, basal-like BRCA subtypes are associated with a poor prognosis [32]. Currently, numerous studies are investigating immune therapies for BRCA, especially basal-like subtypes, though only a minority of patients still appear to respond to this form of therapy. In addition, little is known about the underlying mechanisms of treatment efficacy [33]. The regulatory mechanism of lncRNA in TIME has become an exciting research topic [34]. Therefore, the role of these five lncRNAs was further verified in regard to their biological functions like immunity.

The underlying role of lncRNAs as immune-related prognostic markers remains unclear in BRCA. In the present analysis, the five prognostic immune-related lncRNAs were found to be more reliable indicators in predicting prognosis with a high AUC value (>0.73). In order to detect the viability of the model in a clinical setting, the five immune-related lncRNAs were compared to the clinical features of BRCA patients through a univariate and multivariate COX analysis. As a result, the prognostic model of the five immune-related lncRNAs may contribute in inhibiting the malignant development of BRCA.

lncRNAs participate in multiple biological processes of cancer, including cell cycle [35], DNA repair [36], and glycolysis [37]. The GSEA-based identification of hallmarks and immunologic signature gene sets served was essential in this study. Moreover, the five immune-related lncRNAs were observed to mediate glycolysis, oxidative phosphorylation, and MYC signaling targets. Additionally, immunologic signatures showed that they were also involved in the downregulation of CD8+ T cells and CD4+ Th1 cells, inducing Treg cell upregulation. Evidence revealed that some lncRNAs played a role in tumor immunity, such as the innate immune response and immune cell infiltration [38, 39]. lncRNA Sros1 facilitates innate immune responses by IFN-*γ*-mediated [40], and lncRNA MIR155HG is associated with immune infiltration and immune checkpoint molecule expression in multiple cancers [41]. Similarly, the heterogeneity of TME is very high, and the type and number of immune cells vary greatly among different BRCA types [42]. Risk scores of the five lncRNAs were used to predict their relationship with infiltrating immune cells. Furthermore, the five immune-related lncRNAs were found to be negatively correlated with immune cell infiltration (CD4+ T cells, CD8+ T cells, B cells, dendritic cells, macrophages, and neutrophils) in BRCA, suggesting that the five immune-related lncRNAs play crucial roles in immune infiltration in BRCA.

The advantage of this study is that the proposed model is based on breast cancer novel immune-related data sets as well as high-throughput sequencing data. The ImmLnc datasets are lncRNAs with immune pathway-related activities obtained from TCGA. Combined with clinical information, immune-related lncRNAs as an independent prognostic indicator were obtained. In addition, in order to assess the accuracy of the risk model, both clinical features and breast cancer cell validation were used. Finally, the role of the model in respect to the immune microenvironment was analyzed. Undoubtedly, this study may provide valuable insight into clinical applications for antitumor immunotherapy. Meanwhile, considering that the expressions of the five lncRNAs were also validated in BRCA cells, further verification is necessary to confirm the predictive immune ability in varied BRCA subtypes.

## Figures and Tables

**Figure 1:** Overall flow chart of the present study.

**Figure 2:** (a) Differentially expressed lncRNAs between breast tumors and normal breast tissues identified in the TCGA database. (b) Intersection of differential lncRNAs in the TCGA database and ImmLnc gene sets.

**Figure 3:** Forest plot of hazard ratios shows the prognosis-related value of immune-related lncRNA.

**Figure 4:** (a) Risk score and (b) survival status of the high-risk and low-risk groups. (c) The heat map of expression profile of the five immune-related lncRNAs.

**Figure 5:** Kaplan-Meier survival curve of BRCA patients between the low-risk group and the high-risk group.

**Figure 6:** The five lncRNA expressions were detected by qRT-PCR in BRCA cells and normal breast cells. ^∗^*p* < 0.05, ^∗∗^*p* < 0.01, and ^∗∗∗^*p* < 0.001.

**Figure 7:** Multiple immune-related lncRNAs were associated with clinical characteristics (^∗^*p* < 0.05, ^∗∗^*p* < 0.01, and ^∗∗∗^*p* < 0.001; ns: no relevance). Relationship between immune-related lncRNAs and (a) clinical stage, (b) T-stage, (c) M-stage, (d) N-stage, and (e) age.

**Figure 8:** ROC curve: the AUC for risk score, age, gender, grade, and TNM stage of the total survival risk score were calculated.

**Figure 9:** Several cancer hallmarks and immunologic characteristics regulated *via* the immune-related lncRNAs: (a) glycolysis, (b) oxidative phosphorylation, (c) MYC targets, (d) naive CD4 T cells versus stimulated CD4 Th1 cells down, (e) CD8 T cells down, and (f) Treg cells up.

**Figure 10:** Relationships between the immune-related lncRNA risk scores and infiltration abundances of six types of immune cells: (a) CD4 T cells, (b) CD8 T cells, (c) B cells, (d) dendritic cells, (e) macrophages, and (f) neutrophils.

**Table 1:** The results of multivariate Cox regression coefficients.

lncRNA	Coefficients	HR	HR 95% low	HR 95% high	*p* value
C6orf99	0.154	1.166	1.011	1.345	0.035
LINC00987	-0.188	0.829	0.713	0.964	0.015
SIAH2-AS1	-0.200	0.819	0.724	0.926	0.001
LINC01010	-0.184	0.832	0.741	0.933	0.002
ELOVL2-AS1	-0.160	0.841	0.788	0.910	0.009

**Table 2:** Univariate and multivariate analysis of BRCA.

Variables	Univariate analysis				Multivariate analysis			
	HR	HR 95% low	HR 95% high	*p* value	HR	HR 95% low	HR 95% high	*p* value
Age	1.032	1.017	1.047	<0.001	1.030	1.015	1.045	<0.001
Stage	2.134	1.688	2.698	<0.001	1.637	0.974	2.750	0.063
T	1.519	1.224	1.885	<0.001	1.015	0.743	1.385	0.927
M	6.608	3.710	11.772	<0.001	1.094	0.469	2.553	0.836
N	1.656	1.380	1.989	<0.001	1.136	0.854	1.513	0.381
Risk score	1.769	1.494	2.095	<0.001	1.476	1.224	1.781	<0.001

## Data Availability

The [data type] data used to support the findings of this study are available from the corresponding author upon request.
